# An Autotuning Cable-Driven Device for Home Rehabilitation

**DOI:** 10.1155/2021/6680762

**Published:** 2021-02-11

**Authors:** Jhon F. Rodríguez-León, Betsy D. M. Chaparro-Rico, Matteo Russo, Daniele Cafolla

**Affiliations:** ^1^Instituto Politécnico Nacional-CICATA Querétaro, Querétaro (Qro.) 76090, Mexico; ^2^Biomechatronics Lab, IRCCS Neuromed, Pozzilli (IS) 86077, Italy; ^3^Faculty of Engineering, University of Nottingham, Nottingham NG81BB, UK

## Abstract

Out of all the changes to our daily life brought by the COVID-19 pandemic, one of the most significant ones has been the limited access to health services that we used to take for granted. Thus, in order to prevent temporary injuries from having lingering or permanent effects, the need for home rehabilitation device is urgent. For this reason, this paper proposes a cable-driven device for limb rehabilitation, CUBE^2^, with a novel end-effector (EE) design and autotuning capabilities to enable autonomous use. The proposed design is presented as an evolution of the previous CUBE design. In this paper, the proposed device is modelled and analyzed with finite element analysis. Then, a novel vision-based control strategy is described. Furthermore, a prototype has been manufactured and validated experimentally. Preliminary test to estimate home position repeatability has been carried out.

## 1. Introduction

The access to healthcare services has been significantly limited during the COVID-19 emergency. As face-to-face visits and therapies are reserved to those in need of urgent and essential care, home therapy is preferred when possible. Unfortunately, physical rehabilitation is usually performed by a physiotherapist in one-to-one sessions with a patient. In order to reduce the risk of exposure to infectious diseases such as COVID-19, technologies to enable home rehabilitation are sorely needed to allow patients to perform intensive exercises without visiting hospitals or clinics. Physical therapy and rehabilitation have become inaccessible resources during this pandemic. Thus, Want et al. proposed after-stroke neurorehabilitation therapies that could be carried out at home [1], as they cannot be offered to patients after stroke on the same scale than before. Conversely, the global economic crisis caused by the COVID-19 pandemic will significantly influence industrial robot sales in 2020, as more and more industries move towards digitalization and automation. The adoption of robotic and teleoperated systems will increase worldwide, creating a unique opportunity for robotic-assisted rehabilitation and home-based telerehabilitation [2], which have been mostly developed in research settings rather than commercialized up to now because of a lack of demand.

Several teleoperated medical robotic systems can telemonitor a patient's condition from home [3]. These systems are based on audiovisual teleconferencing, virtual reality, biofeedback, and haptic robotic therapy devices, and the patient gets instructions from a therapist to work alone at home [4]. While most of these systems are under development, a few of them are already commercially available. For example, H-Man [5, 6] is a portable arm rehabilitation robot that helps patients to carry out robot-aided therapy at home. H-Man allows to perform repeated movements recovering motion functionalities lost due to an injury or illness [7]. Another solution, mirror therapy (MT), is proposed in [8]. MT utilizes a mirror that reflects the movement of an unaffected limb and gives the illusion of movement of the affected limb. MERLIN, described in [9], is a robotic telerehabilitation system developed to offer neurorehabilitation at home and it is composed of the ArmAssist (AA) cost-effective robotic system-based games for patients' engagement and training assessment.

Teleoperated systems for physical rehabilitation support face several performance challenges during home rehabilitation, such as the need for adaptability in the difficulty grade of the training, which includes hardware setup, trajectory configuration, resistance settings, and exercise timing [10]. Furthermore, all these rehabilitation devices require a homing position strategy and autotuning in order to avoid the presence of a skilled operator during setup and rehabilitation and enable the autonomous usage of the device by the patient.

The use of cable-driven system has increased in the last few years due to their versatility and advantages, particularly in physical rehabilitation [11–21]. Cable-driven parallel robots replace the rigid links with cables to control the motion of the end-effector (EE), giving a lightweight body and thus making them inherently safe to users because of their low inertia and negligible moving masses [22]. Furthermore, cable-driven mechanisms offer other advantages with respect to rigid link system: high load capacity, stability and smooth motion, larger workspace, undemanding maintenance, low manufacturing costs, easy transportability, lower power consumption, and customizable for a wide range of patients with different anthropometric sizes [23, 24].

In order to support the home rehabilitation for upper and lower extremities during the COVID-19 emergency, this paper proposes a cable-driven device for home rehabilitation, CUBE^2^, that is an evolution of the CUBE (Cable-driven device for Upper and lower limB Exercising) design introduced in [25, 26]. CUBE is a 5-degree-of-freedom (DoF) parallel manipulator with a cable-driven architecture based on six cables, characterized by a fixed frame with adaptable geometry. The EE is shaped as a double ring that is worn as a wristband by the user, and it has been designed with dimensions that are suitable for both upper and lower extremity rehabilitation. The trajectories performed by CUBE can be adapted to different exercises and its cable-driven design makes it inherently safe in human/robot interactions [26]. The CUBE device can be built with commercial aluminum profiles and 3D printed link connectors. As such, it is characterized by a lightweight structure that is easy to set up and operate in both clinical and home environments for both predetermined and customized exercises. However, the original CUBE design could self-calibrate when turned on. Moreover, when a rehabilitation exercise finished with the EE in a different position than the home position, the original CUBE needed to be manually reset to the home position. The mentioned issues made the setup of exercising difficult for the patient without a skilled operator nearby.

Therefore, an autotuning capability is added to the novel CUBE^2^ design, which is also equipped with an improved EE. In this paper, we introduce this novel design and characterize it with its kinematics. A finite element analysis is carried out to compare the performance of the original EE to the novel one. In addition, to identify the initial position of the EE at startup, the control algorithm has been improved from the one of the original CUBE design, which used motors with incremental encoders; the new control strategy includes autotuning for self-calibration. Finally, the manufacturing of the new prototype is described, and laboratory experiments are carried out to validate the novel design. Thanks to the improvements in both control strategy, which includes autotuning based on image processing [27], and EE architecture, the CUBE^2^ device is user-friendly and can be easily used at home for limb rehabilitation without advanced training.

## 2. Conceptual Design of a Novel End-Effector

The CUBE EE was designed to work with a fixed orientation, and it was characterized by three cables connected to an upper connection point and three cables connected to a lower connection point, as illustrated in Figure 1. Therefore, only two connection points were placed on the EE. This configuration limited the controlled rotation of the EE as the fixed connections could generate limited moments. To improve the control over the orientation of the EE, the CUBE^2^ EE has been designed with three distinct connection points in both the upper and lower sections of the EE, so that a unique connection point is used for each of the six cables, as in Figure 2. This novel design allows a fully controlled rotation of the EE, with an improved stress distribution and transmission of the force along the cables. In Figure 3(a), a picture of the original CUBE is shown, whereas in Figure 3(b) a CAD model of the CUBE^2^ device is shown, including the proposed novel EE.

## 3. Kinematic Analysis

The kinematic equations of the CUBE^2^ device are set up by including the novel end-effector (EE) configuration. The upgraded design consists of two frames whose relative motion is controlled by pulling and releasing six cables. The larger frame (“fixed frame”) is fixed to the ground during operation and consists of a triangular prism with height equal to *2h* and radius of the circle circumscribed to the base equal to *r*_0_ (see Figure 4(a)). The smaller frame (“end-effector”), meant to guide the patient's limb, is composed of a central ring-shaped body that is fixed on the patient's wrist or ankle and two triangular-shaped platforms distant 2*d* from each other with cable attachments equally spaced at a radius of *r*_*H*_, as per Figure 4(b). The six extremities of these two frames are connected with cables whose length is actuated by six motors located on the fixed frame.

The behaviour of this design can be described by a parallel kinematic model, following the scheme in Figure 4. The following hypotheses are used to model the cables:

1. The cables are always kept in tension during operation
2. The attachment point of each cable is fixed in position but unconstrained in orientation, thus behaving as a spherical joint
3. The varying length of the cable can be modelled as an actuated prismatic joint

With reference to the fixed frame coordinate system, centered on A_0_, the geometry of the fixed frame is defined as follows:

(1) A00=0;0;0,Ai0=r0cos2iπ3;r0sin2iπ3;−h, for i=1,2,3,Ai0=r0cos2iπ3;r0sin2iπ3;h, for i=4,5,6.

Similarly, with reference to the EE coordinate system, centered on B_0_, the geometry of the end-effector is defined as

(2) BiH=rHcos2iπ3;rHsin2iπ3;−d, for i=1,2,3,BiH=rHcos2iπ3;rHsin2iπ3;d, for i=4,5,6,B00=x;y;z ,B0H=0;0;0.

The transformation between the fixed coordinate system and the EE coordinate system can be described with a translation and a rotation as

(3) tH0=B00−A00,TH0=RH0tH001×311×1,

where ^0^**t**_**H**_ represents the displacement vector between the origins of the coordinate systems, ^0^**R**_**H**_ is the rotation matrix between the two frames, and ^0^**T**_**H**_ is the corresponding transformation matrix. Therefore, it is possible to obtain the length of the cables by writing loop-closure equations as

(4) li=Bi0−Ai0=RH0BiH+tH0−Ai0, for i=1,…,6,

(5) $$\begin{array}{c} l_{i}=\left\|l_{i}\right\|,\;\text{for }i=\left\{1,\ldots ,6\right\}. \end{array}$$

By computing the length of the cables as a function of the EE pose, equations (4) and (5) can be used to solve the inverse kinematic problem of the proposed device, thus enabling its motion control.

## 4. Finite Element Analysis

To analyze the performance of both original and novel end-effector (EE) and understand their behaviour during their performance, a finite element method (FEM) analysis has been carried out. For a suitable discretization for the analysis of cables behaviour during exercising, pulling forces have been computed for each cable in both original and novel EE configurations starting from the known torque of each motor as

(6) $$\begin{array}{c} F=\frac{\tau }{l\;\sin\;\theta }, \end{array}$$

where *F* is the pulling force, *τ* is the motor torque, *l* is the length of the cable, and *θ* is the angle between the cable and the plane of the EE face that is parallel to the triangular face of the frame. As an additional fixture to both scenarios, cables are fixed to the motors in their extremities.

For both EEs' FEM simulation, the average weight of a human arm of 37 N [28] has been applied to the wrist band. The simulation considers also the contribution of gravity. Cables have been considered as made of Dyneema® fiber whose characteristics are reported in Table 1. EEs have been considered as made of acrylonitrile butadiene styrene (ABS), whose characteristics are listed in Table 2. The connection between the cables and the EEs made using commercial components has been considered as made of alloy steel, whose characteristics are listed in Table 3. The characteristics of the mesh used for both simulation scenarios are summarized in Table 4.

As stress analysis criterion for both scenarios, the von Mises stress criterion has been used as a measure that accounts for all six stress components of a general 3D state of stress. The von Mises stress function *σ*_VM_ can be expressed by three stress components in the following form:

(7) $$\begin{array}{c} \sigma_{\text{VM}}=\sqrt{\frac{{\left(\sigma_{1}-\sigma_{2}\right)}^{2}+{\left(\sigma_{2}-\sigma_{3}\right)}^{2}+{\left(\sigma_{3}-\sigma_{1}\right)}^{2}}{2}}, \end{array}$$

where *σ*_1_, *σ*_2_, and *σ*_3_ are the three principal stresses acting on *x*-, *y*-, and *z*-axes of the cable body. The von Mises stress is a nonnegative, scalar stress measure that evaluates elastoplastic properties. This number function represents a stress magnitude, which can be compared against the yield strength of the material in order to determine whether or not failure by yielding is predicted.

### 4.1. Original CUBE End-Effector Simulation

The original EE is composed of 2 bodies, one that slides into another, and these bodies are connected to three cables on the top using a single point and three cables on the bottom using a single point.  Figure 5 shows a rendering of the model used for the FEM simulation.

For the original EE simulation scenario, equation (6) is solved to find the applied pulling forces to each cable *l*=536.11 mm while *θ*=36.04*þ*°, resulting in an applied pulling force along each cable of *F*=7.44 N.

Stress distribution results are shown in Figure 6. In this simulation scenario, it is clear that no stresses in the model exceed the material yield strength for all the components. The maximum computed stress value is reached on the wrist housing along the cables and at the junction between the cable and EE. The stress reaches a maximum, namely, of 5.616 × 10^6^ N/m^2^ and of 2.129 × 10^−2^ N/m^2^. As expected, the stresses are distributed along the ring and are concentred in the right part in the middle of the ring, making it a possible failure point together with the single cable connection points.

### 4.2. Novel CUBE^2^ End-Effector Simulation

The novel EE is composed of 2 bodies, symmetrical apart from the wrist housing. The number of points of connection changes from two (one for three cables on the top and one for three cables on the bottom) to six (one for each of the six cables). Furthermore, each connection has idle degrees of freedom (DoF) along its *Z*-axis, as per Figure 4.  Figure 7 shows a rendering of the model used for the FEM simulation.

In the novel EE simulation scenario, equation (6) is solved to find the applied pulling forces to each cable *l*=393.76 mm while *θ*=37.10*þ*° giving an applied pulling force along each cable of *F*=10.42 N.

Stress distribution results are shown in Figure 8. Also, in this simulation scenario, no stresses in the model exceed the material yield strength for all the components. The maximum computed stress value is reached on the wrist housing along the cables and at the junction between the cable and EE. The stress reaches a maximum, namely, of 3.082 × 10^5^ N/m^2^ and of 6.974 × 10^−1^ N/m^2^. As expected, the stresses are distributed along the two parts of the ring and are concentred in the right part in the bottom part. Furthermore, it is important to notice that, in each cable connection, the stress is distributed, creating circular propagation that vanishes without creating problem in the junctions.

When compared to the original CUBE EE, the novel CUBE^2^ EE eliminates stress concentrations in the middle part of the ring that could be a possible failure zone. Furthermore, in the novel EE, the stress is distributed symmetrically, making it stiffer for the considered applied loads. It is important to notice that the novel proposed EE configuration also improves the admissible tension along the cables from 7.44 N to 10.42 N, an important improvement for a better therapy performance.

## 5. Prototype Manufacturing

After checking the feasibility of the novel proposed design, a prototype has been manufactured. The geometrical parameters of the CUBE^2^ and its end-effector (EE) structure are shown in Table 5.

Six 12 V DC motors with a 1 : 150 reductor radio and encoder have been chosen for the actuation system of CUBE. The motors are connected to pulleys to drive the cables. Moreover, tensioners have been manufactured to prevent the cable from sagging and knotting around pulleys, as shown in Figure 9(a). The EE has been produced with additive manufacturing [29, 30] and the use of a bearing with a diameter of 8 mm to allow free rotation as in Figure 9(b). By using 3D printing, the prototype can be both lightweight and low cost, and it can be made with either virgin or recycled materials to achieve the desired properties [31, 32]. The controller cabinet is composed of an Arduino Mega board that is connected to three L298N drivers. Each L298N allows speed and direction control of two DC motors at the same time. The L298N voltages range from 5 V DC to 35 V DC, and the maximum current is 2 A. The power supply generates 12 V DC and a maximum current of 5 A. Two voltage regulators adjust the voltage from 12 V DC to 3.3 V DC to supply the encoders of the motors. Five fuses of 2 A are used for overcurrent protection as in Figure 10. The CUBE^2^ structure has been manufactured by using 20 mm × 20 mm aluminum profiles and 3D printing technology for the 60° profile connectors (Figure 11).

The upgraded CUBE includes a module for autotuning composed of a C920 PRO HD WEBCAM camera [33]. The autotuning strategy is presented in Section 6. The camera is located on the upper part of the upgraded CUBE structure at a height of 75 mm. The module is attached to two points of the CUBE structure to be easily removed and to allow easy transportation. The upgraded CUBE including the module for autotuning is shown in Figure 12, the CUBE weight is 8 kg, and thanks to the additive manufacturing technologies used, the manufacturing price of the prototype is less than US$1000.

## 6. Control Strategy

The main concerns when using a rehabilitation robot are safety, user-friendliness, and repeatability of the trajectory. The manual calibration of the original CUBE design required a skilled operator to manually find the home position of the device every time the device is turned on with the end-effector (EE) in a configuration different from the home position. Therefore, the aim of the novel control strategy is to embed an autotuning strategy to automatically find the home position of the EE. The autotuning is required since each trajectory must start and end at a predefined home position, as the nonlinearity of the kinematic equations prevents the system from performing correctly when starting from a different configuration. Furthermore, a control strategy that includes autotuning is required to restore the home position if the device turns off unexpectedly during operation. The novel strategy here proposed is based on marker detection through image processing. The marker detection strategy is shown in the flowchart in Figure 13. The autotuning algorithm has been developed in Python and is based on real-time image analysis. Furthermore, the proposed algorithm has been embedded and communicates in real time with the graphical user interface (GUI) of the CUBE^2^ prototype.

By using the procedure illustrated in Figure 13, the proposed algorithm for marker detection calculates the coordinates of the EE from an image frame. The steps for marker detection have been numbered from 1 to 3. Step (1) captures a frame using the camera to allow marker identification as in Figure 14(a). Step (2) consists of colour identification of the used marker. Therefore, the image frame is converted into grey colour scale as in Figure 14(b) and the marker area is identified through contour analysis as in Figure 14(c). In Step (3), the centroid positions in real-world size of the marker are calculated with respect to the image reference frame, defined as *a*. The centroid position is composed of ^**a**^**X**_**j**_ and ^**a**^**Y**_**j**_ coordinates where **j**=**hp** when the EE is placed at home position and **j**=**cp** when the EE is located outside the home position as in Figure 14(d). By storing the coordinates of the marker with the EE at home position, namely, ^**a**^**X**_**hp**_ and ^**a**^**Y**_**hp**_, and calculating the current coordinates of the marker ^**a**^**X**_**cp**_ and ^**a**^**Y**_**cp**_, the current marker coordinates with respect to the Cartesian fixed reference frame named ^0^**X**_**a**_ and ^0^**Y**_**a**_ can be calculated using the following equation:

(8) Xa0 =Xhpa−Xcpa,Ya0=Yhpa−Ycpa.

The marker distance with respect to the camera is estimated using the triangle similarity method described in [34]. The marker distance ^**b**^**Z**_**j**_ is estimated with respect to a reference frame at the camera named *b*. According to the similarity method, the focal length **C**_**f**_ of the camera can be estimated using the marker width in pixels (**P**), the marker width in real-world sizes (**L**), and the distance ^**b**^**Z**_**hp**_ of a marker with respect to the camera. The perceived focal length **C**_**f**_ of the camera can be expressed as follows:

(9) Cf=PZhpbL.

Once **C**_**f**_ is calculated, it can be used as constant data to calculate the distance ^**b**^**Z**_**cp**_ of the marker when the EE is located outside the home position. From equation (9), the current distance ^**b**^**Z**_**cp**_ of the marker in real-world sizes can be evaluated as follows:

(10) Zcpb=CfLP.

Consequently, the ^0^**Z**_**b**_ coordinate of the marker can be estimated as follows:

(11) Zb0=Zhpb−Zcpb+d2.

The marker information (^0^**X**_**a**_, ^0^**Y**_**a**_, ^0^**Z**_**b**_) when the EE is at home position, as well as the current marker information when the EE is outside of home position, can be used for autotuning within the control. A red square marker has been placed on the EE. The square shape information can be accessed using only homography [35]. Using square shapes naturally indicates 4 possible orientations offering more information than shapes such as the circles that have no natural orientation indicators [36, 37]. In the upgraded CUBE, the marker width in real-world sizes (**L**) is 70 mm, the distance from the camera to the EE at home position (^**b**^**Z**_**hp**_) is 1080 mm, the marker width in pixels (**P**) is 42.49 pixels at home position, and the perceived focal length **C**_**f**_ is 650.1 mm at home position.

The control strategy for the actuation is based on a PID control algorithm with a closed-loop control using encoder data and marker information as feedback.  Figure 15(a) shows a scheme of the autotuning strategy where (^0^**X**_**a**_, ^0^**Y**_**a**_, ^0^**Z**_**b**_) are calculated using the marker detection strategy when the EE is located at a current position. Then, these Cartesian parameters are sent to the inverse kinematic of the CUBE to calculate the motor angles (^0^*θ ***cp**_**i**_). Therefore, the position error of the motors (^0^*θ ***e**_**i**_) is calculated using the subtraction of the (^0^*θ ***hp**_**i**_) and ^0^*θ ***cp**_**i**_, where ^0^*θ ***hp**_**i**_ correspond to motor angles when the EE is located at home position. By using ^0^*θ ***e**_**i**_ and the motor angles measured by the encoders (^0^*θ*_**Enc**_), the PID control moves the EE to home position. When ^0^*θ ***hp**_**i**_=^0^*θ ***cp**_**i**_, the encoders are reset, and the rehabilitation trajectory execution is enabled.

Figure 15(b) shows a scheme of the strategy for rehabilitation trajectory execution, where the motor angles (^0^*θ ***in**_**i**_) are calculated using desired rehabilitation trajectories (^0^**X**_**n**_, ^0^**Y**_**n**_, ^0^**Z**_**n**_) as inputs in the inverse kinematic. Therefore, the motor angles are sent to the PID algorithm to locate the EE at the desired position.

The upgraded CUBE control has been integrated to a user-friendly GUI for easy operation, as shown in Figure 16. The user interface allows to perform four programmed exercise trajectories for upper arm rehabilitation that were proposed for the original CUBE in [26]. In addition, it is possible to use the autotuning strategy when the EE is located outside the home position. A text box informs the user the status of the system. Moreover, an emergency button allows the user to stop the system if required.

## 7. Experimental Tests

Preliminary tests have been carried out to estimate the repeatability of the system in the home position when using the autotuning strategy. The aim of the experiments is to measure the ability of the mechanism to reach the home position from a set of poses by using the proposed autotuning strategy. Thus, six critical poses have been identified within the mechanism workspace to test the proposed algorithm. These poses consist of the limit positions reached by the end-effector (EE) along the axes *X*, *Y*, and *Z* in positive and negative quadrants. The repeatability for *X*, *Y*, and *Z* (*Rx*, *Ry*, and *Ry*) has been computed using equations from the Norm ISO 9283 [38] as follows:

(12) $$\begin{array}{c} lx_{i}=x_{i}-\bar{X},\\ ly_{i}=y_{i}-\bar{Y},\\ lz_{i}=z_{i}-\bar{Z},\\ \bar{Lx}=\frac{1}{n}\sqrt{\sum_{i=1}^{n}lx_{i}^{2}},\\ \;\bar{Ly}=\frac{1}{n}\sqrt{\sum_{i=1}^{n}ly_{i}^{2}},\\ \bar{Lz}=\frac{1}{n}\sqrt{\sum_{i=1}^{n}lz_{i}^{2}},\\ Sx=\sqrt{\frac{\sum_{i=1}^{n}{\left(lx_{i}-\bar{Lx}\right)}^{2}}{n-1}},\\ Sy=\sqrt{\frac{\sum_{i=1}^{n}{\left(ly_{i}-\bar{Ly}\right)}^{2}}{n-1}},\\ Sz=\sqrt{\frac{\sum_{i=1}^{n}{\left(lz_{i}-\bar{Lz}\right)}^{2}}{n-1}},\\ Rx=\bar{Lx}+3Sx,\\ Ry=\bar{Ly}+3Sy,\\ Rz=\bar{Lz}+3Sz, \end{array}$$

where *x*_*i*_, *y*_*i*_, and *z*_*i*_ are the reached positions by the EE; $\bar{X},\bar{Y}$, and $\bar{Z}$ are the average of the reached positions; *lx*_*i*_, *ly*_*i*_, and *lz*_*i*_ are the errors; $\bar{Lx}$, $\bar{Ly}$, and $\bar{Lz}$ are the average of the squared errors; and *Sx*, *Sy*, *Sy*, and *Sz* are the standard deviations of the reached positions.

To measure the reached positions of the EE *x*_*i*_, *y*_*i*_, and *z*_*i*_, a distance sensor has been selected as optimal for validating the self-calibration [37]. Thus, a laser sensor, the Parallax Laser Range Finder [39], has been implemented within an experiment layout, as shown in Figure 17. To measure *x*_*i*_, the laser sensor has been placed in front of the axis *X* of the mechanism as shown in Figure 17(a). To measure *y*_*i*_, the laser sensor has been placed in front of the axis *Y* of the mechanism as shown in Figure 17(b). To measure *z*_*i*_, the laser sensor has been placed above the mechanism module as shown in Figure 17(c).

Table 6 shows the estimated mean square errors and their averages, the standard deviation, and the repeatability results for *X*, *Y,* and *Z*, as in similar characterizations in [40, 41]. The measured home position repeatability is 6.53% (normalized on prototype height), in line with the manufacturing and assembly tolerances of the components of the prototype, and can be markedly improved by using a high precision manufacturing process. New strategies for camera calibration can also be implemented to improve image processing and determine the influence of environmental lighting on marker detection precision [42]. In addition, further mechanical solutions for cable tensioning can improve the error produced when the cables are rolled up and down.

## 8. Conclusions

In this paper, a novel device for limb rehabilitation is proposed. The proposed design is an evolution of the CUBE design that includes a novel end-effector for improved wearability, mechanical performance, and motion control, as well as self-calibrating capabilities thanks to a new vision-based autotuning strategy to restore the home position after operation and reset pose errors. The new prototype is characterized with a kinematic model and analyzed through finite element analysis. Then, a low-cost prototype is presented with its manufacturing process through 3D printing and commercial components. The hardware and software for the new control system are then detailed, and experimental tests validate the performance of the proposed CUBE^2^ design.

In conclusion, the new user-friendly interface, the improved end-effector design, and the autotuning capabilities allow patients to use the proposed device autonomously from home, thus enabling rehabilitation training without the need for a physiotherapist nearby. In future developments, the components of the system will be manufactured with improved mechanical tolerances to improve repeatability. Furthermore, a new strategy for camera calibration will be implemented to improve image processing in dim lighting, and additional mechanical tensioners will be added to the prototype for a better dynamic performance.

## Figures and Tables

**Figure 1:** Original CUBE EE connection points. (a) Front view. (b) Connection details.

**Figure 2:** Novel CUBE^2^ EE connection points. (a) Front view. (b) Connection details.

**Figure 3:** Evolution of CUBE. (a) A picture of the original CUBE prototype. (b) CAD model of CUBE^2^, including the proposed novel EE.

**Figure 4:** Kinematic diagram of the proposed design with main parameters. (a) Side view. (b) Top view.

**Figure 5:** Original end-effector (EE) rendering within a FEM (finite element method) scenario.

**Figure 6:** Original CUBE EE FEA von Mises stress distribution. (a) Top view. (b) Bottom view.

**Figure 7:** Novel EE FEM scenario rendering.

**Figure 8:** Novel EE FEM von Mises stress distribution. (a) Top view. (b) Bottom view.

**Figure 9:** CUBE system actuation. (a) DC motor with encoder. (b) Novel EE.

**Figure 10:** Controller box details.

**Figure 11:** Upgraded CUBE prototype.

**Figure 12:** Upgraded CUBE with autotuning calibration module.

**Figure 13:** Marker detection strategy.

**Figure 14:** Identification of the EE. (a) Capture frame. (b) Grayscale image transformation. (c) Square area contours and centroid identification. (d) Centroid tracking.

**Figure 15:** Upgraded CUBE control. (a) Autotuning strategy. (b) Strategy for rehabilitation trajectory execution.

**Figure 16:** Control interface of CUBE.

**Figure 17:** Home position repeatability of CUBE. (a) *X* coordinate. (b) *Y* coordinate. (c) *Z* coordinate.

**Table 1:** Dyneema® fiber for the cables.

Yield strength	7.00 × 10^7^ N/m^2^
Tensile strength	3.60 × 10^9^ N/m^2^
Elastic modulus	1.00 × 10^9^ N/m^2^
Poisson's ratio	0.50
Mass density	980 kg/m^3^
Shear modulus	3.00 × 10^9^ N/m^2^

**Table 2:** ABS characteristics for end-effectors.

Yield strength	45.00 N/m^2^
Tensile strength	3.00 × 10^7^ N/m^2^
Elastic modulus	2.00 × 10^9^ N/m^2^
Poisson's ratio	0.39
Mass density	1020.00 kg/m^3^
Shear modulus	3.19 × 10^8^ N/m^2^

**Table 3:** Alloy steel characteristics for the connections of the commercial components.

Yield strength	6.20 × 10^8^ N/m^2^
Tensile strength	7.24 × 10^8^ N/m^2^
Elastic modulus	2.10 × 10^11^ N/m^2^
Poisson's ratio	0.28
Mass density	7700.00 kg/m^3^
Shear modulus	7.90 × 10^1^ N/m^2^

**Table 4:** Mesh characteristics for modelling.

Mesher used	Curvature-based mesh
Jacobian points	4 points
Maximum element size	6.4103 mm
Minimum element size	1.000 mm

**Table 5:** Geometrical parameters.

Dimension	Value (mm)
*r*_0_	375
*r*_*h*_	63.5
*h*	325
*d*	148

**Table 6:** Repeatability of the prototype (normalized on prototype height).

Coordinates	*x* (mm)		*y* (mm)		*z* (mm)	
Variables	$\bar{Lx}$	*Sx*	$\bar{Ly}$	*Sy*	$\bar{Lz}$	*Sz*
Result	5.80	2.26	10.9	6.81	10.16	8.62
Repeatability	*Rx*=±1.83%		*Ry*=±4.03%		*Rz*=±4.80%	

## Data Availability

The numeric data used to support the findings of this study are included within the article.
